RETRACTED

# Protective Effect of Triphala against Oxidative Stress-Induced Neurotoxicity

**DOI:** 10.1155/2021/6674988

**Published:** 2021-04-07

**Authors:** Wanchen Ning, Simin Li, Jokyab Tsering, Yihong Ma, Honghong Li, Yuezhu Ma, Anthony Chukwunonso Ogbuehi, Hongying Pan, Hanluo Li, Shaonan Hu, Xiangqiong Liu, Yupei Deng, Jianlin Zhang, Xianda Hu

**Affiliations:** ^1^Department of Conservative Dentistry and Periodontology, Ludwig Maximilian University of Munich, Goethestrasse 70, Munich 80336, Germany; ^2^Stomatological Hospital, Southern Medical University, Guangzhou 510280, China; ^3^Laboratory of Cell and Molecular Biology, Beijing Tibetan Hospital, China Tibetology Research Center, 218 Anwaixiaoguanbeili Street, Chaoyang, Beijing 100029, China; ^4^Department of Neurology, Graduate School of Medical Sciences, Kumamoto University, Kumamoto, Japan; ^5^Peking University Third Yanqing Hospital, 28 East Shuncheng St., Yanqing District, Beijing 110229, China; ^6^Faculty of Physics, University of Münster, Wilhelm-Klemm-Straße 9, Münster 48149, Germany; ^7^School of Dentistry, University of Michigan, 1011 N University Ave, Ann Arbor, MI 48109, USA; ^8^Department of Cranio/Maxillofacial Surgery, University Clinic Leipzig, Liebigstr. 12, Leipzig 04103, Germany; ^9^Innovation Center Computer Assisted Surgery (ICCAS), Leipzig University, Semmelweisstraße 14, Leipzig 04103, Germany; ^10^Department of Neurosurgery, Taian Central Hospital, Taian City, Shandong Province 271000, China

## Abstract

**Background:**

Oxidative stress is implicated in the progression of many neurological diseases, which could be induced by various chemicals, such as hydrogen peroxide (H_2_O_2_) and acrylamide. Triphala is a well-recognized Ayurvedic medicine that possesses different therapeutic properties (e.g., antihistamine, antioxidant, anticancer, anti-inflammatory, antibacterial, and anticariogenic effects). However, little information is available regarding the neuroprotective effect of Triphala on oxidative stress.

**Materials and Methods:**

An *in vitro* H_2_O_2_-induced SH-SY5Y cell model and an *in vivo* acrylamide-induced zebrafish model were established. Cell viability, apoptosis, and proliferation were examined by MTT assay, ELISA, and flow cytometric analysis, respectively. The molecular mechanism underlying the antioxidant activity of Triphala against H_2_O_2_ was investigated dose dependently by Western blotting. The *in vivo* neuroprotective effect of Triphala on acrylamide-induced oxidative injury in *Danio rerio* was determined using immunofluorescence staining.

**Results:**

The results indicated that Triphala plays a neuroprotective role against H_2_O_2_ toxicity in inhibiting cell apoptosis and promoting cell proliferation. Furthermore, Triphala pretreatment suppressed the phosphorylation of the mitogen-activated protein kinase (MARK) signal pathway (p-Erk1/2, p-JNK1/2, and p-p38), whereas it restored the activities of antioxidant enzymes (superoxide dismutase 1 (SOD1) and catalase) in the H_2_O_2_-treated SH-SY5Y cells. Consistently, similar protective effects of Triphala were observed in declining neuroapoptosis and scavenging free radicals in the zebrafish central neural system, possessing a critical neuroprotective property against acrylamide-induced oxidative stress.

RETRACTED

**Conclusion:**

In summary, Triphala is a promising neuroprotective agent against oxidative stress in SH-SY5Y cells and zebrafishes with significant antiapoptosis and antioxidant activities.

## 1. Introduction

Oxidative stress is implicated in the progression of many inflammatory and malignant diseases, including neurodegenerative disease (such as Alzheimer's disease [1], Parkinson's disease [2], mild cognitive impairment [3, 4], and vascular dementia [5]), as well as oral disorders like dental caries, periodontal disease [6, 7], oral mucositis [8], and oral cancer [9]. The severe or prolonged oxidative stress is mainly induced by the excessive production of reactive oxygen species (ROS), which causes DNA damage, oxidative proteins, and peroxidation of lipids and thereby triggers cell apoptosis [10, 11]. ROS is composed of superoxide anion (^·^O_2_^−^), hydrogen peroxide (H_2_O_2_), and hydroxyl radicals (OH^·^) [12], of which H_2_O_2_ is a culprit, destroying neurons, and thus is widely used as a stimulant of neutral cells to establish an *in vitro* oxidative injury model [13, 14]. In addition, acrylamide, a vinyl monomer formed in high-temperature foods [15], is applied as a neurotoxin in various cell and animal models for its overproduction of ROS. For instance, acrylamide was suggested to induce cell apoptosis in human neuroblastoma SH-SY5Y cells [16] and promote neurotoxicity in the zebrafish model [17].

Triphala, or *‘Bras Bu gSum Thang*'in Tibetan, is a well-recognized Ayurvedic medicine consisting of dried fruits of three plant species, including *Emblica officinalis* (family *Euphorbiaceae*), *Terminalia bellirica* (family *Combretaceae*), and *Terminalia chebula* (family *Combretaceae*). Modern studies have shown that Triphala has many properties, including antihistamine, antioxidant, antitumor, anti-inflammatory, antibacterial, antiviral, antifungal, and anticariogenic effects [18, 19]. In addition, Triphala has been investigated to be effective in treating many types of cancers and oral diseases, including prostate cancer [20], pancreatic cancer [21], colon cancer [22], and gynecological cancers [23], as well as periodontal diseases [24]. Regarding Triphala's neuroprotective ability, a research group from Taiwan has revealed the protective effect of *Terminalia chebula* extracts on a neuron-like rat pheochromocytoma (PC12) cell line [25, 26]. Thus, it is of note that Triphala has many possibilities to possess neuroprotective property. However, despite the recent report, current information regarding the neuroprotective effect of Triphala is still limited. Thus, the present study is aimed at investigating Triphala's neuroprotective property against oxidative stress-induced damage *in vitro* and *in vivo*.

RETRACTED

## 2. Materials and Methods

### 2.1. Cell Culture

Human neuroblastoma (SH-SY5Y) cells were provided by China Infrastructure of Cell Line Resource. SH-SY5Y cells were cultured in Dulbecco's modified Eagle medium (DMEM) (Corning), supplemented with 10% fetal bovine serum (FBS) (Corning) and 1% penicillin-streptomycin (Beyotime Biotechnology Inc., Nantong, China). The cells were incubated at 37°C under a humidified atmosphere of 5% carbon dioxide.

### 2.2. MTT Assay for Cell Viability Analysis

SH-SY5Y cells were seeded in 96-well plates (CoStar, USA) separately at a density of 4,000 cells per well. Triphala extract power (AL1675; Dabur India Ltd., Alwar, India) was prepared and diluted in the same way as our previous study [23, 27]. Firstly, to determine the optimal concentrations of Triphala and H_2_O_2_, higher concentrations (0.08, 0.4, 2, 10, 50, and 250 *μ*g/mL) and lower concentrations (0.014, 0.041, 0.12, 0.37, 1.11, 3.33, and 10 *μ*g/mL) of Triphala were applied to treat SH-SY5Y cells for 48 h. Meanwhile, cells were treated with 300, 400, 500, 600, 700, and 800 *μ*mol/L of hydrogen peroxide (H_2_O_2_) for 20 h, separately. Then, cell viability was measured using 3-[4,5-dimethylthiazol-2-yl]-2,5-diphenyl-tetrazolium bromide (MTT) assay (Boster Biological Technology Company, Wuhan, Hubei, China). Briefly, each well was incubated with 10 *μ*L of MTT solution for 4 h at 37°C, added with 110 *μ*L formazan solvent, and the absorption at 490 nm was measured using a microplate reader (Beijing Pulang New Technology Co., Beijing, China).

Next, the neuroprotective effect of Triphala on H_2_O_2_ toxicity was estimated by preincubating cells with increasing concentrations (0.014, 0.041, 0.12, 0.37, 1.11, 3.33, and 10 *μ*g/mL) of Triphala for 24 h and then challenging the cells with 400 *μ*mol/L H_2_O_2_ for an additional 20 h. Cells treated without either H_2_O_2_ or Triphala were considered as blank control, while the H_2_O_2_-induced injury cell model, in which only H_2_O_2_ was added, was regarded as model control. After the drug intervention, cell viability was determined using the MTT assay as described above and the percentage of cell viability was calculated as follows: viability (%) = (OD_experiment_ − OD_blank_)/(OD_model_ − OD_blank_) × 100%. The percentage of the protective effects was calculated; thus, protective effects (%) = 1 − viability (%).

RETRACTED

### 2.3. ELISA Assay for Cell Apoptosis Analysis

The Cell Death Detection Enzyme-Linked Immunosorbent Assay (ELISA) Plus Kit (Roche Diagnostics, Basel, Switzerland) was applied to examine the apoptosis inhibition activity of Triphala as our previous study [23]. Briefly, the cells were seeded and cultured using the same method described above. SH-SY5Y cells in the logarithmic growth phase were seeded in 96-well plates and pretreated with different concentrations (0.37, 1.1, and 3.3 *μ*g/mL) of Triphala for 24 h. Then, cells were treated with 400 *μ*mol/L H_2_O_2_ for an additional 20 h. The setup of the blank control and model control was the same as above. After the drug intervention, the cells were collected and resuspended in lysis buffer and the lysate was centrifuged to remove the intact nuclei. The supernatant containing cytoplasmic histone-associated DNA fragments was transferred into a streptavidin-coated microplate and was then incubated with immunoreagent and substrate for quantitative immunoassay. The OD value was determined at 405 nm using a microplate reader, and the fold increase of DNA fragmentation, reflecting the number of programmed cell deaths, was calculated as absorbance of treated cells/absorbance of negative control cells.

### 2.4. Flow Cytometric Analysis

Flow cytometry assays were processed using monoclonal antibody Ki-67 and Annexin V/propidium iodide (PI) double staining, to evaluate the degree of proliferation apoptosis, as in our previous study [23]. Briefly, SH-SY5Y cells were seeded into 6-well plates (Nest Biotech., China) at a density of 1 × 10^5^ cells per well. After pretreatment with different concentrations (0.37, 1.1, and 3.3 *μ*g/mL) of Triphala for 24 h, the cells were treated with 400 *μ*mol/L H_2_O_2_ for an additional 20 h. Then, the cells were harvested by trypsinization, incubated with −20°C in absolute ethanol, washed, and resuspended in cell staining buffer. Subsequently, cells were fixed and the nuclear membrane was permeabilized using Foxp3/Transcription Factor Staining Buffer Set (eBioscience Inc., San Diego, CA) before staining with anti-Ki67 antibody (Miltenyi Biotec, Bergisch Gladbach, Germany) at 4°C for 1 h. To detect the apoptosis, cells were incubated using the FITC Annexin V Apoptosis Detection Kit with PI (Dojindo Molecular Technologies Inc.), at room temperature for 15 min. Afterwards, the fluorescent staining was detected and analyzed using a flow cytometer (BD Biosciences, San Jose, CA). The mean fluorescent intensity for Ki-67 was calculated using FlowJo VX software (Tree Star Inc., Ashland, OR).

RETRACTED

### 2.5. Western Blot Analysis

SH-SY5Y cells were seeded in the 10 cm Petri dishes with a density of 5 × 10^5^ cells per dish. Firstly, the cells were pretreated with increasing concentrations (0.37, 1.1, and 3.3 *μ*g/mL) of Triphala for 24 h and stimulated with 400 *μ*mol/L H_2_O_2_. The blank control and model control were established as described above. Then, the cultured cells were harvested by centrifugation and fractionated using the Nuclear and Cytoplasmic Protein Extraction Kit (Beyotime Biotechnology Inc., Nantong, China) following the manufacturer's instruction with the supplement of protease inhibitor cocktail and phosphatase inhibitor cocktail, offered by Sigma-Aldrich Corp. (St. Louis, MO). The protein concentrations were determined using the Pierce BCA Protein Assay Kit (Thermo Fisher Scientific, Waltham, MA). The total or nuclear proteins were separated by SDS-PAGE electrophoresis, transferred to a nitrocellulose membrane, and then incubated with monoclonal antibodies, including phospho-p44/42 mitogen-activated protein kinase (MAPK) extracellular signal-related kinase (ERK)1/2. (Thermo Fisher), phospho-c-Jun amino-terminal kinases (JNK)1/2 (Thermo Fisher), and phospho-p38 MAPK, superoxide dismutase 1 (SOD1), and catalase, which were purchased from Cell Signaling Technology (Danvers, USA). Afterwards, rabbit anti-mouse secondary antibody (Abcam, Cambridge, UK) and goat anti-rabbit secondary antibody (Abcam) were attached and expression levels of proteins were detected by chemiluminescence using a Pierce ECL Plus Western Blotting Substrate (Thermo Fisher).

### 2.6. Zebrafish Embryos

The wild-type AB strain of zebrafishes (*Danio rerio*) were obtained from Hunter Biotechnology (Hangzhou, China). The zebrafishes were maintained in the 28°C reverse osmosis water, incubating with 200 mg/L instant sea salt and 50–100 mg/L CaCO3, at an electrical conductivity of 450~550 *μ*S/cm and a pH of 6.5–8.5. The embryos used in this study were generated by natural pairwise mating.

### 2.7. *In Vivo* Maximum Tolerated Concentration (MTC) of Triphala

A total of 270 wild-type AB strain zebrafishes were randomly selected at 1 day postfertilization (dpf), and 30 zebrafishes per well were plated in 6-well plates (Nest Biotech., China). Acrylamide stock (L2028046; Aladdin, Shanghai, China) was dissolved with DMSO into 1 mol/L, 30 *μ*L of which was then added into 3 mL fish water, reaching the final concentration (10 mmol/L). Triphala was prepared as described above. Prepared acrylamide was applied to establish a zebrafish neuroapoptosis model. Then, to explore the maximum tolerated concentration (MTC) of Triphala, we treated the acrylamide-stimulated zebrafishes together with different concentrations of 3 mL Triphala (0.123, 0.370, 1.11, 3.33, 10.0, 30.0, and 90.0 *μ*g/mL) at the same time, for 24 h. The control group was incubated with neither Triphala nor acrylamide, while 10 mM acrylamide only stimulated the model group.

RETRACTED

### 2.8. *In Vivo* Neuroprotective Effect of Triphala

A total of 240 wild-type AB strain zebrafishes were randomly selected at 1 dpf, and 30 zebrafishes per well were plated in 6-well plates. Control and model groups were established as described above. Five different concentrations of 3 mL water-soluble Triphala (0.123, 0.370, 1.11, 3.33, and 10.0 *μ*g/mL) were applied to treat the 10 mM acrylamide-induced fishes at the same time. Glutathione (GSH) powder (SLCF2362; Sigma-Aldrich, Shanghai, China) was diluted into 615 *μ*g/mL, and 3 mL GSH was used to stimulate the acrylamide-induced fishes together, regarded as a positive control group to compare the effects of Triphala. Then, the eight groups of fishes were incubated at 28°C for 24 h. Then, the fishes were stained with acridine orange (AO) (494-38-2, Sigma, China). After that, ten zebrafishes from each group were randomly selected, which were observed and imaged using a fluorescence microscope (VertA1; Shanghai Tucson Vision Technology Co., China). The mean fluorescence intensity was analyzed using NIS-Elements D 3.20 image software. The statistical analysis of the fluorescence intensity was used to evaluate the neuroprotective efficacy of Triphala.

### 2.9. *In Vivo* Antioxidant Effect of Triphala

A total of 240 wild-type AB strain zebrafishes were randomly selected at 1 dpf, and 30 zebrafishes per well were plated in a 12-well plate (Nest Biotech., China). Control and model groups were established as described above. Five different concentrations of 3 mL water-soluble Triphala (0.123, 0.370, 1.11, 3.33, and 10.0 *μ*g/mL) and 615 *μ*g/mL GSH were applied to treat the acrylamide-induced fishes together. Meanwhile, 2 mL E3 medium with ROS-specific fluorescent substrate (CM-H2DCFDA) (C6827/2146733; Invitrogen, USA) was added into each well. Subsequently, the fishes and medium were transferred into a 96-well plate (CoStar, USA) and incubated for 20 h at 28°C (protected from light). Next, the plate was scanned with the multifunctional enzyme marker (Spark; Tecan, Switzerland) and each group's fluorescence was measured. Finally, the fluorescence value of each group was collected and analyzed using SPARKCON TROL Dashboard software. The fluorescence value was used to evaluate the ability of Triphala in scavenging free radicals.

RETRACTED

### 2.10. Statistical Analysis

All in vitro data were represented as means ± SDs of a minimum of 3 independent experiments. Statistical analyses were carried out by one-way ANOVA, with Bonferroni correction, via SPSS Statistics 26.0 software. A *p* value < 0.05 was considered to be statistically significant.

## 3. Results

### 3.1. Optimal Concentration of Triphala and Hydrogen Peroxide (H_2_O_2_) in SH-SY5Y Cells

In order to determine the optimal concentration of Triphala applied in the subsequent experiments, the proliferation rate of various concentrations of Triphala was firstly measured using MTT assay. Among the higher concentrations (from 0.08 to 250 *μ*g/mL) of Triphala, only 50 and 250 *μ*g/mL Triphala significantly decreased cell viability, with the proliferation rates of −17.84% and −56.38% (*p* < 0.05), compared to blank control (see Figure 1(a)). However, lower concentrations (from 0.014 to 10 *μ*g/mL) of Triphala promoted cell viability in SH-SY5Y cells, of which 0.37, 1.11, and 3.33 *μ*g/mL Triphala dramatically enhanced the proliferation rates to 142.55%, 183.12%, and 226.80% (*p* < 0.05) (see Figure 1(b)). By virtue of these results, pretreatment with low concentrations of Triphala (from 0.014 to 10 *μ*g/mL), especially 0.37, 1.11, and 3.33 *μ*g/mL, was considered as optimal to examine its neuroprotective effect against H_2_O_2_-induced damage.

Aimed at determining the optimal concentration of H_2_O_2_ to exert neurotoxicity, the apoptosis rate of various concentrations of H_2_O_2_ was measured using an MTT assay. Relative to 300, 400, 500, 600, 700, and 800 *μ*mol/L (*μ*M) of the H_2_O_2_ apoptosis rate was upregulated to 30.14%, 47.65%, 63.53%, 80.41%, 80.36%, and 79.78%, respectively (see Figure 1(c)). Based on the above, the half-maximal inhibitory concentration (IC50) of H_2_O_2_ was 400 *μ*mol/L; thereby, stimulating 400 *μ*mol/L H_2_O_2_ for 20 h was considered as optimal and applied in subsequent experiments.

### 3.2. Neuroprotective Effect of Triphala on SH-SY5Y Cells

Aimed at determining Triphala's neuroprotective effect on H_2_O_2_-induced SH-SY5Y cells, cell viability was measured by the MTT assay. In a dose-dependent experiment, increasing concentrations of Triphala were applied to preincubate the SH-SY5Y cells which were then treated with H_2_O_2_. Corresponding to 0.014, 0.041, 0.12, 0.37, 1.11, 3.33, and 10 *μ*g/mL Triphala pretreatment, the calculated protective rates were 17.82%, 54.98%, 61.08%, 109.22%, 125.65%, 108.34%, and 61.96%, respectively (see Figure 1(d)). Except the lowest concentration (0.014 *μ*g/mL), other concentrations of Triphala markly (0.041, 0.12, 0.37, 1.11, 3.33, and 10 *μ*g/mL) upregulated the protective rates in the H_2_O_2_-induced SH-SY5Y cells (*p* < 0.05), compared to the model control (see Figure 1(d)). Combined, Triphala played a protective role in attenuating the cell viability loss in SH-SY5Y cells treated with H_2_O_2_.

RETRACTED

### 3.3. Inhibition of Triphala on H_2_O_2_-Induced Apoptosis in SH-SY5Y Cells

ELISA was used to determine the effect of Triphala on H_2_O_2_-induced apoptosis in SH-SY5Y cells. Compared to the model control, the apoptosis inhibitory rates of H_2_O_2_-induced SH-SY5Y cells were significantly upregulated to 22.53%, 23.66%, and 35.45%, by 0.37, 1.11, and 3.33 *μ*g/mL Triphala, respectively (*p* < 0.05) (see Figure 2(a)). The above results suggested an inhibitory effect of Triphala in suppressing the apoptosis stimulated by H_2_O_2_.

### 3.4. Proliferative Effect of Triphala on H_2_O_2_-Induced SH-SY5Y Cells

The cell proliferation rate was evaluated by flow cytometry analysis using the FITC Annexin V Apoptosis Detection Kit. As shown in Figure 2(b), the results revealed a significant reduction of 20.60% in the proliferation rate in SH-SY5Y cells exposed to H_2_O_2_, compared to the blank control. In contrast, 0.37, 1.11, and 3.33 *μ*g/mL Triphala preincubation increased the proliferation rates by 17.93%, 15.11%, and 22.81%, in the H_2_O_2_-induced SH-SY5Y cells (see Figure 2(b)). The results suggested that H_2_O_2_ is an inhibitor, but Triphala is a promoter in the SH-SY5Y cell proliferation.

### 3.5. Investigation of Molecular Pathways

To further determine the neuroprotective mechanisms of Triphala, the expression of p-ERK1/2, p-JNK1/2, p-p38 MAPK, SOD1, and catalase was examined in H_2_O_2_-induced SH-SY5Y cells by Western blotting. Higher levels of p-Erk1/2, p-JNK1/2, and p-p38 and lower levels of SOD1 and catalase were expressed in the model control, relative to blank control (see Figure 2(c)). Furthermore, the degrees of p-Erk1/2 and p-p38 in the H_2_O_2_-induced SH-SY5Y cells were decreased by 0.37 and 1.1 *μ*g/mL Triphala pretreatment (see Figure 2(c)). On the contrary, in comparison with the model control, 3.3 *μ*g/mL Triphala promoted the expression of p-Erk1/2, as well as p-p38 (see Figure 2(c)). As to the p-JNK1/2 content, upregulation of JNK protein was inhibited by Triphala preincubation (0.37, 1.1, and 3.3 *μ*g/mL) in the SH-SY5Y cells exposed to H_2_O_2_ and p-JNK1/2 expression was dramatically attenuated to the lowest level, which is similar to that expressed in blank control (see Figure 2(c)).

Significant upregulation of SOD1 was stimulated by 0.37, 1.1, and 3 *μ*g/mL Triphala pretreatment in the H_2_O_2_H2O2-induced SH-SY5Y cells, relative to model control (see Figure 2(c)). Moreover, 3 *μ*g/mL increased the SOD1 degree to the highest point that is even higher than blank control (see Figure 2(c)). Similarly, higher protein levels of catalase were stimulated by Triphala preincubation (0.37, 1.1, and 3.3 *μ*g/mL) in SH-SY5Y cells exposed to H_2_O_2_, compared to both model and blank controls (see Figure 2(c)). Combined, the three concentrations (0.37, 1.1, and 3 *μ*g/mL) of Triphala applied in the experiment were efficient in restoring the levels of neuroprotective-related proteins in the SH-SY5Y cells exposed to H_2_O_2_.

RETRACTED

### 3.6. MTC of Triphala in the Zebrafish Model

In our study, the MTC of Triphala was determined firstly according to the fish (mammalian) toxicology [28]. The threshold of Triphala should be, on the one hand, high enough to maximize the neuroprotective effect. On the other hand, the preferred concentration would not be too high to induce neurotoxicity [17, 29]. As Table 1 showed, three engagements, 1.11 *μ*M (1/9 MTC), 3.33 *μ*M (1/3 MTC), and 10.0 *μ*M (MTC), were selected as the preferred concentration of Triphala in the following experiment, which promoted better biological phenotypes of the zebrafishes, compared to the model fishes. Otherwise, Triphala of 30.0 and 90.0 *μ*g/mL exerted toxicity and induced worse biological phenotypes of the zebrafishes, leading to a 3.33% (1/30th) mortality of the fishes. Zebrafishes treated with 0.123 and 0.370 *μ*g/mL Triphala performed similarly to the model fishes. Thus, the MTC of Triphala *in vivo* was determined as 10.0 *μ*g/mL.

### 3.7. Triphala Suppressed Acrylamide-Induced Neurotoxicity in the Zebrafish Model

According to the fluorescence intensity, Triphala's *in vivo* neuroprotective effects were observed in the zebrafish model injured by acrylamide. The fluorescence intensity of the control group (4153043 pixels) was significantly lower than that of the model group (10860891 pixels) (*p* < 0.05) (see Figures 3 and 4(a)), indicating that the zebrafish model was successfully established. Also, the fluorescence intensity of the GSH-treated-positive group (4517110 pixels) was significantly lower than that of the model group (*p* < 0.05) (see Figures 3 and 4(a)), suggesting the neuroprotective effects of the GSH on acrylamide. The fluorescence intensity rates of the increasing concentration (0.123, 0.370, 1.11, 3.33, and 10.0 *μ*g/mL) of Triphala were 8611230, 6392234, 4382534, 4313911, and 4155579, respectively. Triphala of 0.123 and 0.370 *μ*g/mL exerted no significant protective effects on zebrafishes exposed to acrylamide (*p* > 0.05) (see Figures 3 and 4(a)). However, decreasing pixels of 1.11, 3.33, and 10.0 *μ*g/mL Triphala were detected, compared to the model group (*p* < 0.05) (see Figures 3 and 4(a)). The findings supported that Triphala, a comparable neuroprotective agent as GSH, inhibited the acrylamide-induced neuroapoptosis in zebrafishes.

RETRACTED

### 3.8. Triphala Scavenged Free Radicals in the Zebrafish Model Exposed to Acrylamide

Based on the fluorescence value, the antioxidative effects of Triphala in vivo were evaluated in the zebrafish model exposed to acrylamide. The fluorescence value of the control group was 1667, which was significantly lower than that of the model group (2363) (*p* < 0.05) (see Figure 4(b)), supporting the practicability of the zebrafish model. Besides, compared to that of the model group, the reduced fluorescence value of the GSH-treated-positive group (124) was measured (*p* < 0.05) (see Figure 4(b)), indicating that GSH is an efficient antioxidant agent in scavenging the free radicals produced by acrylamide. The fluorescence intensity rates of the increasing concentration (0.123, 0.370, 1.11, 3.33, and 10.0 *μ*g/mL) of Triphala were 858, 816, 716, 746, and 1168, respectively. Except for 10.0 *μ*g/mL Triphala, other concentrations of Triphala (0.123, 0.370, 1.11, and 3.33 *μ*g/mL) significantly decreased the level of free radical, relative to that of the model group (*p* < 0.05) (see Figure 4(b)). The findings suggested Triphala's comparable antioxidant efficiency as GSH in scavenging the free radicals in zebrafish exposed to acrylamide.

## 4. Discussion

Herewith, we investigated the antioxidant and neuroprotective aspects of Triphala using an *in vitro* H_2_O_2_-induced SH-SY5Y cell model and an *in vivo* acrylamide-induced zebrafish model. Our MTT, ELISA, and flow cytometric results indicated that Triphala could attenuate the cytotoxic effects of H_2_O_2_ by promoting cell proliferation and inhibiting cell apoptosis. Moreover, the underlying mechanisms were analyzed by Western blotting, demonstrating that pretreatment of Triphala upregulated antioxidant enzymes (SOD1 and catalase) and suppressed MAPK (p-Erk1/2, p-JNK1/2, and p-p38) activation, which in turn exerted its neuroprotective effects on inhibiting cellular apoptosis against oxidative damage. Consistently, *in vivo* immunofluorescence staining evidenced the neuroprotective role of Triphala against the neurotoxicity induced by acrylamide in zebrafishes.

The cell viability level and proliferation rate are recognized as good indicators of cell health [30]. In our study, H_2_O_2_ exposure induced apoptosis of SH-SY5Y cells by decreasing cell viability and inhibiting cell proliferation, consistent with previous reports [14, 31]. Possessing antioxidant properties, our previous study suggested the antitumor effect of Triphala on inhibiting the proliferation and increasing the apoptosis in many cancer cell lines [23]. In contrast, one fruit of Triphala (*Terminalia chebula* extract) was investigated by another two studies, suggesting its neuroprotective effects on enhancing cell viability in H_2_O_2_-treated PC12 cells [25, 26]. Our experiment first evaluated Triphala's neuroprotective effect on H_2_O_2_-induced SH-SY5Y cells to the best of our knowledge. Triphala dose-dependently increased the proliferative and protective rates of SH-SY5Y cells exposed to H_2_O_2_, while Triphala markly attenuated the H_2_O_2_-induced increase in apoptosis. Consistently, Triphala's protective activity is similar to the neuroprotective peptide Orexin-A in increased proliferation in SH-SY5Y cells induced by H_2_O_2_ [14]. In general, the findings overall indicated that Triphala plays a neuroprotective role in alleviating the H_2_O_2_-induced neurotoxicity.

RETRACTED

Notably, based on immunofluorescence staining results, Triphala was evidenced as a comparable neuroprotective potent as GSH, decreasing the acrylamide-induced toxicity in the central neural system of zebrafish. In line with the previous reports, our study confirmed that acrylamide could contribute to neuroapoptosis [32] and promote the free radicals in zebrafishes. GSH is determined as a known antioxidant that plays an essential role in balancing the oxidative stress in brain cells [32]. Besides, reduced GSH has been implicated in many neurological diseases, such as Parkinson's disease [33], Alzheimer's disease [34], epilepsy [35], and Huntington's disease [36]. In consistant with these reports, GSH application in the current study inhibited the neuroapoptosis and production of free radicals in zebrafish exposed to acrylamide. Similarly, Triphala possessed equivalent neuroprotective and antioxidant effects as GSH. Our findings first demonstrated that Triphala (especially 1.11 and 3.33 *μ*g/mL) could decline neuroinjury and scavenge the free radicals in the zebrafish central neural system, exerting a critical neuroprotective property against acrylamide-induced oxidative stress.

Additionally, Triphala's underlying antioxidant mechanisms were also determined in a dose-dependent experiment by Western blotting through measuring neuroprotective-related proteins' expressions. Two major cellular antioxidant enzymes, SOD1 and catalase, can scavenge the ROS products to control the antioxidant system [37]. Recent studies reported that Triphala effectively attenuated oxidative stress via SOD1/catalase restoration both *in vitro* and *in vivo* [38]. For instance, Triphala extracts were able to quench free radicals by inducing SOD and catalase against bacteria [39]. Meanwhile, Triphala could increase the SOD and catalase expressions in the selenite-induced cataract model [40]. Furthermore, due to its antioxidant potential, Triphala restored the levels of SOD and CAT in a rat model of colitis [41] and arthritis [42]. In line with the above evidence, our finding revealed that H_2_O_2_ exposure decreased expressions of SOD and catalase in SH-SY5Y cells, whereas the reductions were enhanced by Triphala (0.37, 1.1, and 3 *μ*g/mL) pretreatment. Moreover, higher concentrations of Triphala tend to be more efficient as it promoted the expression to a level even higher than the blank control. The restoring activities of SOD and catalase in the H_2_O_2_ injury model indicated the neuroprotective role of Triphala in antioxidant processes via activating the SOD1/catalase clearance pathway.

RETRACTED

Furthermore, ERKs, p38 MAPKs (p38), and JNKs the three well-known MAPK signal pathways, were investigated in the Triphala-induced antioxidant activities [43]. Recognized as the essential mediators, MAPK signaling pathways underlining the neural diseases are attracting more and more attention. Several studies have validated oxidative stress results in neural damage via MAPK signal cascades [43, 44]. For example, a significant increase in the phosphorylation of ERK1/2, JNK1/2, and p38 MAPK protein was detected in the ischemic penumbra rat model with middle cerebral artery occlusion and reperfusion [45]. Consistent with the previous findings, the present study has proven that H_2_O_2_ promoted apoptosis through upregulating the phosphorylation of p-Erk1/2, p-JNK1/2, and p-p38 in SH-SY5Y cells. More importantly, our finding firstly demonstrated that Triphala attenuated the levels of p-Erk1/2, p-JNK1/2, and p-p38 in the H_2_O_2_-induced SH-SY5Y cells, indicating its antioxidant and neuroprotective properties against oxidative stress. Interestingly, in a dose-dependent experiment, unlike the fact that 0.37 and 1.1 *μ*g/mL Triphala significantly suppressed the activation of p-Erk1/2, p-JNK1/2, and p-p38, 3 *μ*g/mL Triphala downregulated the p-JNK1/2 level. In contrast, it upregulated the contents of p-Erk1/2 and p-p38. As mentioned, it is worth noting that Triphala is meanwhile proposed to be prooxidant in promoting the apoptosis of cancer cells by releasing ROS productions [38]. Oral administration of 50/100 mg/kg Triphala significantly induced apoptosis in Capan-2 cancer cells through ROS generation, associated with increased expression of p53 and ERK [21]. In the normal cells, ROS usually is low; however, the level rises in the cancer cells, which crosses the threshold and forces the cell into apoptosis [46]. Considering that SH-SY5Y cell is a human neuroblastoma cell line, Triphala's prooxidant activity in our experiment is a possibility, being supported by our investigation indicating that 50 and 250 *μ*g/mL Triphala suppressed cell proliferation.

RETRACTED

However, some limitations still existed in this study. First, the major focus is put on the antioxidant activities of Triphala, whereas, as mentioned above, the application of high or low concentrations of Triphala is likely to exert opposite effects on the proliferation rate of cancer cells, accounting for its prooxidant ability in combating tumors. These observations led to the hypothesis that the pleiotropic functions of Triphala on regulating oxidative stress may depend on various conditions. Furthermore, as a multi-ingredient formulation, Triphala consists of three fruit herbal medicines and hundreds of components, the majority of which are polyphenols and their bioactive metabolites, such as gallic acid, quinic acid, teresautalic acid, chebulinic acid, corilagin, salicin, ethyl gallate, and methyl gallate [47–50]. Therefore, one point of further study should explore pharmacological mechanisms of the critical compounds with various concentrations in regulating antioxidant activities using different cell models. Second, few reports on the neuroprotective effects of Triphala are cognitive and only major antioxidant genes and vital signaling pathways were investigated in this study. Thus, the identification of the compound-target gene network is of great importance. Bioinformatics analysis, such as gene ontology enrichment analysis, functional pathways analysis, and target protein/miRNA interaction analysis, could facilitate a better understanding of the possible ingredients, targets, and mechanisms. Third, up to now, although a few clinical trials on Triphala have been done, such as gingivitis (NCT01898000) and periodontal disease (NCT01900535), most of the studies are done in animals and *in vitro* models; thus, more *in vivo* and clinical studies are needed in multiple conditions prior to its applicability.

It is important to note that this present research's findings also have a transfer value for future clinical use. Recently, there is an upsurge in the areas related to applying Triphala as an alternative therapy in various diseases due to its gifted therapeutic activity and minimal or no side effects. Neutralizing oxidative stress is core in the treatment of both neurodegenerative diseases and oral disorders. By that, Triphala's antioxidant and protective effects revealed in this study will also be pertinent to examine how Triphala plays a vital role in dentistry. For instance, Triphala was identified as an antibacterial and anti-inflammatory agent in treating periodontal diseases, with comparable chlorhexidine efficacy but without any detected side effect [24]. Moreover, Triphala could be applied as a root canal irrigant in treating primary endodontic infections, considering the high toxicity of the efficient irrigant (sodium hypochlorite). In addition, possessing the inhibitory activity against PMN-type collagenase, Triphala could be an alternative medicine of doxycycline in healing periodontal destruction, without side effects. Furthermore, other potential applications of Triphala in the oral cavity are noteworthy, such as wound healing of oral mucosa and regeneration in hard and soft tissues. Nevertheless, the detailed molecule mechanisms under these benefits of Triphala also necessitate investigations in the context of dentistry in well-designed preclinical studies.

RETRACTED

## 5. Conclusion

In summary, the current *in vitro* study firstly indicated the neuroprotective effect of Triphala on attenuating H_2_O_2_-induced apoptosis in SH-SY5Y cells via restoration of the antioxidant enzymes (SOD1 and catalase) and suppression of the MAPK (p-Erk1/2, p-JNK1/2, and p-p38) activation. Furthermore, Triphala was evidenced as a comparable neuroprotective potent as GSH *in vivo*, which declined neuroapoptosis and scavenged free radicals in the zebrafish central neural system, possessing a critical neuroprotective property against acrylamide-induced oxidative stress. Consequently, Triphala might be a potential therapeutic agent to treat neurodegenerative diseases associated with oxidative stress.

## Figures and Tables

**Figure 1:** Effects of Triphala and hydrogen peroxide (H_2_O_2_) on cell viability in SH-SY5Y cells. (a) Cell viability promotion effect of Triphala on SH-SY5Y cells. SH-SY5Y cells were treated with higher concentrations (0.08, 0.4, 2, 10, 50, and 250 *μ*g/mL) of Triphala for 48 h. (b) Proliferative effect of Triphala on SH-SY5Y cells. SH-SY5Y cells were treated with lower concentrations (0.014, 0.041, 0.12, 0.37, 1.11, 3.33, and 10 *μ*g/mL) of Triphala for 48 h. (c) Cytotoxic effect of H_2_O_2_ on SH-SY5Y cells. SH-SY5Y cells were treated with different concentrations (300, 400, 500, 600, 700, and 800 *μ*mol/L) of H_2_O_2_ for 20 h. (d) Protective effect of Triphala on H_2_O_2_-induced apoptosis in SH-SY5Y cells. SH-SY5Y cells were pretreated with increasing concentrations (0.014, 0.041, 0.12, 0.37, 1.11, 3.33, and 10 *μ*g/mL) of Triphala for 24 h and then exposed to 400 *μ*mol/L of H_2_O_2_ for 20 h. The data are expressed as mean ± SD (*n* = 3). ^∗^*p* < 0.05 as compared to control.

RETRACTED

**Figure 2:** Effect of Triphala on hydrogen peroxide (H_2_O_2_)-induced apoptosis in human neuroblastoma SH-SY5Y cells. SH-SY5Y cells were preincubated by 0.37, 1.11, and 3.33 *μ*g/mL Triphala for 24 h and then exposed to 400 *μ*M H_2_O_2_ for 20 h. In the control group, cells were not treated with either H_2_O_2_ or Triphala. In the model group, only H_2_O_2_ was added into cells, without Triphala incubation. (a) ELISA kit was used to determine the apoptosis inhibitory effect of Triphala on H_2_O_2_-induced SH-SY5Y cells. (b) Flow cytometry analysis was applied to evaluate the cell proliferation rate. (c) Western blotting was performed to determine the degrees of the neuroprotective proteins (p-Erk1/2, p-p38, p-JNK1/2, SOD, and catalase) in the H_2_O_2_-induced SH-SY5Y cells with/without Triphala pretreatment. The blots shown are representative of three independent experiments. *β*-Actin was used as a loading control. Data are expressed as mean ± SD (*n* = 3). ^∗^*p* < 0.05 as compared to control.

**Figure 3:** Representative photographs of the brain area (central nervous system) of the zebrafish model. The control group was incubated with neither Triphala nor acrylamide. The model group was only exposed to 10 mM acrylamide for 24 h. Glutathione (GSH) of 615 *μ*g/mL was applied to treat the acrylamide-induced zebrafishes together for 24 h (positive control group). Increasing concentrations (0.123, 0.370, 1.11, 3.33, and 10.0 *μ*g/mL) of Triphala were applied to treat the acrylamide-induced fishes for 24 h at the same time (experiment group). The *in vivo* neuroapoptosis is stained in green and detected with the fluorescence microscope.

**Figure 4:** Effects of Triphala and acrylamide on zebrafishes *in vivo*. (a) The neuroprotective effects of Triphala *in vivo* were evaluated in the zebrafish model injured by acrylamide, according to the fluorescence intensity. Increasing concentrations (0.123, 0.370, 1.11, 3.33, and 10.0 *μ*g/mL) of Triphala, as well as 615 *μ*g/mL glutathione (GSH), were applied to treat the acrylamide-induced zebrafishes together for 24 h. (b) The antioxidative effects of Triphala *in vivo* were evaluated in the zebrafish model exposed to acrylamide, according to the fluorescence value. Increasing concentrations (0.123, 0.370, 1.11, 3.33, and 10.0 *μ*g/mL) of Triphala, as well as 615 *μ*g/mL glutathione (GSH), were applied to treat the acrylamide-induced zebrafishes together for 20 h. Control: zebrafishes incubated with fish water; model: zebrafishes only exposed to acrylamide. The data are expressed as mean ± SD (*n* = 3). ^∗^*p* < 0.05 as compared to control.

RETRACTED

**Table 1:** MTC exploration of Triphala *in vivo*.

Group (*n* = 30)	Triphala concentration (*μ*g/mL)	Number of deaths (tails)	Mortality (%)	Biological phenotypes
Control	/	0	0.00	Normal
Model	/	0	0.00	Pericardial oedema; slight bending of the bodies
Triphala+acrylamide	0.123	0	0.00	Similar to the model
	0.370	0	0.00	Similar to the model
	1.11	0	0.00	Better than the model
	3.33	0	0.00	Better than the model
	10.0	0	0.00	Better than the model
	30.0	1	3.33	Worse than the model
	90.0	1	3.33	Worse than the model

## Data Availability

The data used to support the findings of this study are available from the corresponding author upon request.
